The article "Promoting Environmental Protection through Art: The Feasibility of the Concept of Environmental Protection in Contemporary Painting Art" was published in 2022. Journal: J Environ Public Health.

# Promoting Environmental Protection through Art: The Feasibility of the Concept of Environmental Protection in Contemporary Painting Art

**DOI:** 10.1155/2022/3385624

**Published:** 2022-09-26

**Authors:** Xiangping Zou

**Affiliations:** Pan Tianshou College of Architecture, Art and Design, Ningbo University, Ningbo, 315000 Zhejiang, China

## Abstract

With the development of society and the progress of science and technology, the impact of human beings on the environment is becoming more and more serious but also facing the crisis of resource exhaustion. The frequent occurrence of natural disasters has sounded the alarm to human beings, and people are paying more and more attention to the concept of green ecology. There is a close relationship between people and the environment, the development of industry, and the abuse of resources, so that today's ecological environment has been greatly damaged, people's requirements for the environment are constantly improving, and people's environmental awareness is also increasing. While vigorously strengthening environmental management, the government also put forward the “people-oriented” sustainable development strategy. Along with the development of The Times, the art of graphic design is an important service in the field of the society, serves people, is the service life of important activities, its art function must keep pace with The Times, should not only meet the needs of The Times, and to be able to meet the needs of The Times, and to be able to meet the needs of the market. More should make full use of the function of the design to influence and change the society through design ideas, to advocate environmental protection, to improve people's thinking patterns and values, and to change those production and life styles that deviate from sustainable development. Therefore, this article will discuss and analyze the modern painting from the artistic concept, art education, green environment concept, green design, and so on.

## 1. Introduction

### 1.1. Creation Background of Ecological Painting

Ecological painting is purely hand-painted with materials such as natural plants, plants, and even butterflies according to their shapes, colors, and sizes. It is a kind of art, a kind of culture, and a combination of art. The original work is based on scientific specimens and the beautiful art of embossing. It can satisfy people's thirst for flowers for thousands of years and make it prosperous. It is the best choice for people at home, restaurants, hotels, offices, and shops. It is a sign of social status and upbringing. With the improvement of mechanization, China's economic development speed is getting faster and faster, but due to environmental pollution, some local environmental problems are more and more serious; the government is also paying more and more attention to environmental protection [1], but there is no way to timely solve the environmental problems in cities and villages. There are more and more people on earth, and people are competing with other life for survival. Some people have begun to realize the importance of environmental protection, but their environmental awareness is still in the bud. Although they have been aware of the deterioration of the environment, their quality of life is not good, their environmental awareness is still very low, their confidence in nature is constantly collapsing, and the problem of environmental protection has a long way to go.

### 1.2. The Necessity of Ecological Painting

From the perspective of the whole ecosystem, ecological painting shows people's concern about the ecological balance of nature and themselves, thus arousing people's concern about nature and the surrounding living environment. Reconstruction of underground pipelines in the old city is difficult, and residents have to endure the stench. The sewage and waste from the mink farms are not treated, and the water in the fish ponds has become undrinkable [2].

Villagers are still raising ferrets in the most primitive way [3]. People tend to ignore results, do things without thinking through them, have a hard time thinking about the bigger picture, and have an inert conformity mentality. In the development of contemporary ecological art, oil painting, as an ancient and composed form of expression, can also express the needs of the environment and the public from the perspective of the public. At the same time, ecological painting can also carry out necessary communication with the public [4]. From the perspective of public education, it is easier for both adults and children to understand and participate.

### 1.3. Basic Concepts of Green Design

Green design is an international design trend emerging in the late 1980s. Green design is not only a reflection on the environmental and ecological damage caused by modern science and technology but also a return to the designer's ethics and social responsibility. In the long history of human beings, industrial design has not only provided modern living and living environment for people but also accelerated the consumption of resources and energy and seriously damaged the earth's ecosystem. In particular, the excessive commercialization of industrial design has made design an important medium, which encourages people to carry out unrestricted consumption. No wonder people call “advertising design” and “industrial design” the “primary culprit” of publicizing mass consumption, which has attracted a lot of accusations. In this context, designers must reflect on the responsibilities and roles of industrial designers, so green design comes into being, as shown in Figure 1. “3R” is the basic principle of green design [5]. The reduction principle is to reduce the consumption of matter and energy and the discharge of harmful substances. The reuse principle is to design the product and its parts so that they can continue to be used after treatment. The recycling principle is that the recyclability of materials should be considered in product design.

### 1.4. Psychology of Art

#### 1.4.1. Differences between Art Psychology and General Education Psychology

As psychology exists in pedagogy, it can better enrich itself and thus guide educational activities, as shown in Figure 2. Our goal, then, was to find unique ways to enrich ourselves in art teaching and that came naturally to us [6]. Through comparison, we can see that art psychology is a unique way in art teaching.

The psychology of art is a science that studies artistic creation and human psychology [7]. This is the kind of knowledge that leads to a better understanding of art [8]. Therefore, art education and art education are closely linked. Art psychology is a kind of psychological reconnection, which has strong practicability and can show its application well. In Europe, the development of psychology and physics is particularly prominent in the 19th century, while the development of applied psychology has gone through the baptism of wisdom and history and gradually matured with the development of psychology. In this era, in the world of art, a new and unique discipline emerged, that is, experimental aesthetics.

#### 1.4.2. Characteristics of Educational Psychology

Educational psychology is a scientific field belonging to applied psychology as well as artistic psychology [9]. Educational psychology takes various psychological phenomena in education and teaching as the research object and the change of this phenomenon, as well as the psychological law of the educated people in the environment of “teaching” and “learning” to learn technology and cultivate intelligence and personality. Of course, neither does educational psychology [10]. Therefore, educational psychology is mainly concerned with the cultivation and development of students' psychological characteristics.

The main content of educational psychology is summarized as the following four aspects:

1. Individual psychological differences
2. Formation and rules of technology
3. Psychological characteristics of the educated in mastering technology and techniques
4. Moral cultivation and cultivation of educates

### 1.5. Research Purpose and Significance of Spatial Metaphor

As a new concept, spatial metaphor was proposed by Rakoff and Johnson in 1980. As an academic term, its research is currently limited to language and cognition. Therefore, after reviewing a large number of studies on metaphor and spatial metaphor, the author looked back at Tuymans and the works of several contemporary artists using space as the medium and found many similarities with modern oil painting art. Metaphor can break through our past thinking inertia and construct a new logical relationship for us. Through analogy, projection, and other new perspectives and methods, we can effectively expand our thoughts, so that our thoughts can be better expanded into an unknown abstract world, thus making new connections between our thoughts and feelings. In contemporary art, as an important participation factor, spatial metaphor is increasingly valued by people, but there is no systematic theory to analyze it at present [11]. Secondly, this paper mainly draws lessons from metaphors from other disciplines so that metaphors in contemporary art can be applied to other studies, thus extending metaphors to art.

## 2. Description of the Problem

### 2.1. Status Quo of Ecological Art

Ecological art, ecological photography, ecological film, and so on are gradually rising in China. In the 1990s, Chinese local artists are also trying to go global in the way of contemporary ecological art. In the 21st century, the world has taken the industry by storm [12]. For example, the combination of art and photography and a large number of environmental photography sites like China emerged to take practical action to protect the environment. Ecological photography is a kind of ecological art, which can actively make the audience feel protected and close to nature.

Compared with China, foreign ecological art is more diverse and creative, and artists themselves are also the backbone of environmental NGOs. They persevere and go into the public space through the form of art to promote the importance of environmental protection but also recognize the contribution of art to society and call on the public to actively participate. The painter has a direct involvement in the treatment of environmental problems.

### 2.2. Green Urgency

With the development of science and technology, contemporary design has more space for development and more forms of expression [13], at the same time deep into the level of design thinking, resulting in the change of design concept, namely, depletion and destruction of ozone layer, greenhouse effect, earth overload, destruction of biological chain, reduction of forest vegetation, resource depletion, urban solid waste pollution, sulfur dioxide smog event in Maas Valley of Belgium, London smog event, and Beijing haze event. Human beings originally hope to inspire designers' moral and social responsibility through the perspective of professional self-discipline [14]. Chinese scholars appeal: Design should not be limited to the infinite expansion of commerce and consumption, and the code of conduct of design is the ethics of design. From the perspective of ethics, the design has been comprehensively considered, including the factors of people, environment, and resources, so as to shoulder the historical task of serving the environment with limited resources and healthy development of human beings. Chinese scholars believed that he had to talk to the public and instill a new concept of “fit is good” in the society with the most basic ideas. However, in the past 50 years, in the struggle between ethics and commercial interests, and in today's deteriorating ecological environment, the “humble” working attitude of designers has declared the failure of design ethics. In order to find a way out of survival, people began to take the road of mandatory law, which opened a new era of “green design,” as shown in Table 1.

### 2.3. The Aesthetic Interest of Painting Art

Plagiarism, piecing together the blind imitation of doctrine, results in a variety of not mean neither fish nor fish weird atmosphere. From multifarious vanity to simplicity, from waste of beauty to insistence on the environment, the industry has a responsibility to reverse this vice. As a country with a long history, China's thousand-year civilization has bred a unique outlook on life and ethics. How to integrate the essence of Chinese traditional culture into our design is an important task entrusted to us by The Times. Here, it must be pointed out that the spirit and form of tradition are different; how to grasp its essence, rather than just stay on the surface of simple imitation, this problem is worthy of in-depth discussion and research by the design circles at home and around the world.

### 2.4. Key Issues of Ecological Painting Creation

One of the key points of ecological painting creation is to choose appropriate materials and expressions [15]. Creation requires the selection of a theme closely related to people's life, and the seemingly ordinary theme is properly expressed and highlighted by various means of painting.

The second key is how to explain the relationship between man and nature. From what point of view? But he looked at himself. How to correctly and vividly describe environmental pollution can not only make the audience better understand the relevant knowledge of the environment but also correctly understand the relationship between human and nature and guide the audience to constantly think about what they should do to change this phenomenon. While destroying the environment is protecting the environment, art is art, influencing others from a subconscious point of view, combined with ecological civilization. The third point is to skillfully combine personal experience with ecological creation to make the work more full and full of spirit and meaning, as shown in Table 2.

## 3. State of the Art

### 3.1. Requirements of Ecological Painting Creation

Ecological painting should conform to the basic principles of ecology and environmental science and be combined with facts, be reasonable and well-grounded, and have a good role in environmental education. Also, ecological painting triggers reflections on social, environmental, and human relationships [16]. At the same time, the creation of ecological oil painting should also follow the aesthetic rules of art creation and choose the theme and language close to nature as much as possible, so that the public can better experience its beauty, as shown in Figure 3. Positive emphasis on the beauty of the environment and harmony between man and nature can also be used to describe the real situation of environmental deterioration from a reverse perspective to warn people of the importance of environmental problems. In the creation of ecological oil painting, we should draw lessons from the expression of ways and methods of modern ecological art and, on this basis, innovate it.

### 3.2. Relationship between Sustainable Development Strategy and Green Design Policy

To achieve sustainable development, we must build a recycling society and improve the efficiency of resource and energy reuse.

“Go.” The development of circular economy inevitably needs “reduction, reuse, and recycling” to prevent pollution from the source and build a sustainable production and consumption system, and the key to achieving this goal is to promote green design. Before the 1950s, there were only six international conventions on environmental protection and management, which increased to 16 in the 1970s and more than 100 in the 1980s. Now there are more than 180 international conventions and agreements covering the atmosphere, land, and sea [17]. With the continuous enrichment and expansion of the concept of sustainable development, the formulation and implementation of green design policy also provide a strong impetus for the formation of green design policy in the early 21st century.

However, the strategy of sustainable development is the general direction of mankind and an overall strategic decision. In a particular industry, in the design aspect, there is a great practical value. “Landing” is an important path of sustainable development strategy. Design majors are booming these days, but the price of professional design is high. The lack of values and ethics makes design become a way for developers to grab profits and cheat consumers. Brazzard is in urgent need of new values to reshape its advanced and scientific nature. These two levels are urgent needs for the development of human society and an important driving force for green design policy, as shown in Figure 4. It can be said that the sustainable development strategy points out the direction for the formulation and implementation of green design and provides a strong policy support for it. At the same time, the policy of green design is constantly improving and perfecting the concept of sustainable development.

### 3.3. Painting Art Is the Foundation of Modern Design

Regardless of history, form, language, and other aspects, painting art is the cornerstone of contemporary design. In the practice of brand, painting art also plays a very important role. An Australian industrial design advisory committee in 1998, according to a report, published that a design student should have 10 best skills, namely, “be good at drawing and painting freehand”; this is the basic quality which designers must have; therefore, no manual drawing and design ability are not correct. Painting can promote design thinking and technology, and a simplified icon design is a simple summary and summary of the concrete sketch. In fact, no computer-aided design can replace a sketch on paper.

### 3.4. Painting Art Status Quo

Chinese painting art is good at summary, direct, and casual, through the effect of images to express the artist's aesthetic ideas, the pursuit of levels, and aesthetic interest. Throughout the long history, Chinese painting has been a kind of “noble art” since ancient times. The folk art of the public still exists, but it has not received special treatment [18]. Until today, the traditional Chinese poetry and calligraphy and painting have been well known to people. Among today's Chinese artists, many artists are still inheriting and developing traditional traditions and following the traditions of their predecessors. On the basis of tradition, their artistic styles and characteristics are also constantly developing. The former was the representative of Gu Lin and Jincheng, while the latter was Huang Binhong, Pan Tianshou, and Qi Baishi. Form, shape characteristic, the understanding of Chinese painting and thinking, realistic performance, and shape characteristics constitute the Chinese classical aesthetics and philosophy, in the general observing things, with the size to large and small in see big way, in the observation and understanding in general, and what also not on the surface, are not in a place of rest. Just like the objective images of natural landscapes, flowers, birds, and so on, the observation, understanding, and expression are all consciously connected with human's social consciousness and aesthetic taste, while “freehand brushwork” and “lyric expression” are the expression of the Chinese thought of “unity of nature and man.” In the specific works, attention is paid to the organic combination of poetry and calligraphy, painting, and seal, as well as through the poetic language in the picture; the artist's cognition and expression of society, life, and art are all part of the organic deepening of the theme and picture.

Painting art is rich and colorful; beauty is its essence. Beauty is the basis of human existence and is the basis of continuous progress and development. Western painting focuses on induction and analysis and tends to reason. To analyze the objective world in the way of painting, until modern times, its important works were still widely used in people's daily life, and many painters' works were priced sky-high, but its artistic essence was created for the working people. However, the beauty of artistic discovery is different from the beauty of nature. It is a kind of hazy beauty, which needs more artists to constantly explore and explore! The traditional art of western painting, which can be traced from lines to primitive times, as an independent artistic activity, tries its best to show accurate and flexible purposes. Although it could not get rid of the shackles of Western philosophy, it was at that time due to its precise pursuit of form, as shown in Table 3. Therefore, the scientific relationship with the objective world is relatively close, for example, with the continuous development of painting art, more and more accurate, and more and more realistic, three-dimensional space concept is gradually excavated, and in the art field of painting, there are relatively few art concepts and intelligence.

### 3.5. The Value of Spatial Metaphor in Contemporary Painting Art

#### 3.5.1. Value of Spatial Metaphor in Contemporary Painting Art

Nothingness was used to be an art, but now its size is seen as an art. This is according to an exhibition “The Art of Empty Questions” by American artist Jeanifer Richter. The word “space question” was widely used in The European Renaissance. “Space” is defined as the distance between objects and objects, while the traditional IFL space is represented or served as a background by points, lines, planes, and colors. In the 20th century, the concept of space has been expanded and has a close relationship with psychology, literature, and many other fields. The French phenomenological philosopher Merleau Ponty regarded “empty inquiry” as a universal relation, and he linked “time inquiry“ with the active state of “empty inquiry.” The generation of “empty questioner” originates from the “Lord of space,” which transforms “empty” from a tool of “description”“ to “emotion,” which is reflected in contemporary paintings.

#### 3.5.2. Expansion of Traditional Space Art by Contemporary Space Metaphor

As far back as Greek and Roman times, there was attention to space. Under the influence of “imitation theory,” many excellent painters can well show their pursuit of objects in the use of light and focus. Classical, neoclassical, romantic, realism, and other traditional schools of painting are very high attainments in the simulation of objective things. It is precisely because in the traditional concept, the most important thing is to show real objects, so since the birth of perspective, space has been strictly limited in a series of laws such as big, far and small, near reality, and far and virtual. Through the continuous study of the structure of human vision, painters have been thinking about how to make their works more realistic and more appealing to the audience.

## 4. Results Analysis

### 4.1. Strategic Policy and Structural Environmental Programmes

The strategic policy is based on economic strength, environmental pollution, and technological level [19]. Strategies are guidelines for the development and implementation of environmental protection regulations or codes, as well as social objectives for environmental protection design and cleaner production. It has three main contents sustainable development, environmental protection, and integrated product planning. Environmental action plan and integrated product plan are an important means of sustainable development strategy rather than a dependency [20]. Sustainable development strategy: The action plan will promote the sustainable and efficient use of natural resources, energy, and raw materials, as well as the elimination of hazardous substances and hazardous raw materials from the manufacture and design of products from a source control perspective. Since about 80% of the environmental impacts have been identified at the product design stage, important products should be enhanced with environmental design, such as taxation. The production process is more detailed and cleaner, which is the focus of planning management.

### 4.2. Methods of Green Design

#### 4.2.1. Life Cycle Design Method

Life cycle is a broad concept, which is widely used in politics, economy, environment, technology, society, and other fields. The production of products includes raw material collection, processing, storage, transportation, use, scrap, disposal, and other whole process. The life cycle method is an important approach to green design. This is the test from the beginning of the concept design, from the design, research and development, production, use, disposal, and other whole process to ensure the environmental performance of products. In the process from design to production, the life cycle method is most relevant to “green” products, as shown in Figure 5.

#### 4.2.2. Modular Design Method

One of the most important aspects of green design is modularity [21]. Modular design classifies the function, performance, specifications of the product design, and different selection and combination of functional modules, in order to achieve different functional requirements. Modularization can shorten the design and manufacturing cycle of products, reduce production costs, standardize product varieties, improve quality, and accelerate product updates, as shown in Figure 6. In addition, the product adopts a modular design, is easy to repair, and because of its consistent size, is easy to disassemble, and in the event of local failure, can be quickly replaced and can extend the service life of the product; also, it can be said to kill two birds with one stone.

### 4.3. The Artistic Expression of Painting Improves the Aesthetic Value of Design

Beauty is an emotion in the human heart, a strong thing that awakens the beauty in the deep [22]. This is a man's best wish. Beauty is hidden deep in people's subconscious, unspeakable beauty; artists should draw it well, let people see. This is what a painter should do. The sky in the painting art design should have beauty, beauty not only to the eye, but also the eye. It is a spiritual connection.

### 4.4. Construct the Basic Path of Green Design Policy Implementation

As a kind of public policy, the policy goal of “green design” is long term and complicated, and it must be transformed into specific standards through specific implementation channels: goals or paths to realization. Factors such as science and technology, economy, and culture vary greatly among countries, so the conditions for policy making are also different. Its implementation path has many characteristics. The implementation approach of green design policy in China should be in line with technical feasibility, economic affordability, social acceptance, political acceptance, and implementation of the policy plan. Choose the best strategy by evaluating and choosing the potential risks associated with the path, as shown in Figure 7. The implementation of “green design” mainly includes supporting the research and development of key technologies such as green manufacturing and green production and leading market innovation, establishes incentive mechanism and punishment mechanism, and strengthens the support to small and medium-sized enterprises. The combination of moral guidance and policy incentive constructs the basic mode of green design.

### 4.5. Research and Thinking on the Way of Ecological Art Movement

The connection between traditional artists and the public is broken, and art may be beyond the understanding of ordinary people. We believe that art comes from life, but it is more important than life. The social basis of ecological art can be divided into two kinds: one is natural education institution, the other is natural education institution, and the other is art museum. However, the nature of the two men's societies was quite different. NGO is a public service organization, and the art is often a meeting place for culture-centered social groups. In the exhibition hall, ecological artists focus on the images of animals and humans, using installations, paintings, sculptures, and other art to remind people of the connection between humans and nature, but it is difficult to change their mind. The nature museum, which is open to the public, has the dual attributes of art and science. Physical specimens can also be displayed as a work of art in the museum, attracting more attention and understanding. While appreciating ecological art works, people will spontaneously enter nature to seek peace of mind and the connection between man and nature.

Whether ecological artists care about, improve, and serve the society depends on individual ability and choice. In the contemporary era, ecological artists tend to return to the masses. Ecological art is often the artistic temperament expressed by artists in the social ecological movement. Take Huang Yifeng from Taiwan for example. He uses his environmental art education to encourage more people to participate in the creation of nature and make people realize the importance of the environment. Huang Yifeng's “Cultivation of Natural Observation Talents” and “DIY of Natural Wild Interest” are his experience and practice in ecological art. In the simplest and most direct way, they help more people get spiritual satisfaction in life and also satisfy people's pursuit of nature. Maybe the public's painting and creation techniques are not professional enough, but each person's creativity is unique, the public's concept will gradually change, and people will gradually pay attention to the natural environment.

In contrast, the local natural ecological art movement has a larger space for development. Sun Jun's advocate of “green cross” is the construction of “green,” Beijing's “green cross” to “country” into a “rural,” “ecological,” “ecological,” “environmental protection,” “environmental protection,” “garbage collection,” “classification,” and other “green.” Sun Jun of green cross, in a series of works about rural ecology, has created a real and beautiful picture.

## 5. Conclusions

At present, the global energy is about to be exhausted, and the ecological crisis is imminent. In a sense, this is the issue of environmental protection. Associate designers attempt to awaken “profit seeking” by means of design ethics, so that they wake up and dare to be responsible for their own survival. To solve the current dilemma, the responsibility of protecting the earth's resources and the environment is unrealistic. Categories do not have much time for designers to wake up. What measures should enterprises take under the guidance of sustainable development strategy? Develop flexible green design guidelines and strict environmental regulations to limit the actions of designers. Establishing and perfecting environmental protection system is an urgent problem to be solved at present.

## Figures and Tables

**Figure 1:** Green concept in all aspects of the showe.

**Figure 2:** Knowledge of art psychology and other disciplines.

**Figure 3:** Interdisciplinary and research content.

**Figure 4:** For sustainable development of benign cycle schematic diagram.

**Figure 5:** Green design content and process.

**Figure 6:** Modular design diagram.

**Figure 7:** Material selection principle in green design concept.

**Table 1:** The types and quantities of renewable resources that can be recycled every year in China.

Renewable resources that can be recycled	Iron and steel scrap	Waste paper	Waste tires	Scrap nonferrous	Waste plastics	Other waste materials	A combined
Unit: ten thousand tons	4000	3000	5000	500	600	1000	100 million

**Table 2:** Key issues of ecological painting creation.

The key problem	
Focus on 1	Choose appropriate materials and expressions
Focus on 2	Explain the relationship between man and nature
Focus on 3	Hands-on experience is cleverly combined with ecological creation

**Table 3:** Understanding of contemporary art and its artistic view in basic art education.

The problem		Students	Teachers'
Contemporary art	Do not understand	96%	72%
Focus on contemporary art	Do not focus on	87%	92%
The relationship between contemporary art and schooling	It does not matter	85%	93%
The desire to understand contemporary art	Want to	93%	87%

## Data Availability

The labeled data set used to support the findings of this study is available from the corresponding author upon request.
